The article "Xp11.2 Translocation Renal Cell Carcinoma: Clinical Characteristics and Potential Prognostic Predictors" was published in 2021. Journal: Dis Markers.

# Xp11.2 Translocation Renal Cell Carcinoma: Clinical Characteristics and Potential Prognostic Predictors

**DOI:** 10.1155/2021/5647933

**Published:** 2021-09-01

**Authors:** Jie Dong, Weifeng Xu, Zhigang Ji, Boju Pan

**Affiliations:** ^1^Department of Urology, Peking Union Medical College Hospital, Chinese Academy of Medical Sciences and Peking Union Medical College, Beijing, China 100730; ^2^Department of Pathology, Peking Union Medical College Hospital, Chinese Academy of Medical Sciences and Peking Union Medical College, Beijing, China 100730

## Abstract

**Background:**

Xp11.2 translocation renal cell carcinoma, a rare malignancy, has a higher prevalence in children than in adults. It is relatively indolent in children but manifests with an aggressive course in adults. Clinical characteristics and prognostic studies for adult patients are scarce due to its rarity.

**Methods:**

This retrospective single-center study consecutively enrolled 24 newly diagnosed Xp11.2 translocation RCC adult patients. Clinical presentations were recorded, and baseline laboratory results and follow-up data were collected. Possible risk factors for progression-free survival and overall survival were first scanned with chi-square tests and *t*-tests to compare patients who suffered from progression or death with who did not. Multivariate Cox regression was further utilized to identify independent risk factors.

**Results:**

Twenty-four adult patients (median age 32, range 16-73), with a male-to-female ratio of 1 : 1, was included from April 2010 to March 2020. After follow-up for 35.7 months (+/- months), seven patients died. With univariate analysis, higher C-reactive protein-to-albumin (CRP/Alb) ratio (*p* = 0.028), higher baseline fibrinogen (*p* = 0.006), and presence of distant metastasis (*p* = 0.007) were associated with progression of the disease; higher preoperative fibrinogen (*p* = 0.014) and distant metastasis (*p* = 0.020) were associated with death. With multivariate Cox regression, only baseline fibrinogen level (*p* = 0.001) was identified as an independent risk factor for progression-free survival; meanwhile, fibrinogen level (*p* = 0.048) and distant metastasis (*p* = 0.043) were identified as independent risk factors for survival.

**Conclusions:**

Overall, relatively high CRP/Alb ratios, fibrinogen, and distant metastasis were associated with a poor prognosis of Xp11.2 tRCC adult patients; among them, only baseline fibrinogen levels independently predicted the progression of Xp11.2 tRCC; thus, it may help to identify patients with worse progression or death risk.

## 1. Background

Xp11.2 translocation/TFE3 gene fusion-related renal cell carcinoma (RCC) is a rare and unique subtype of RCC characterized by translocations involving the TFE3 gene [1–3]. It has been classified as a distinct entity in the 2004 World Health Organization renal tumor classification and is now regarded as an important subtype of RCC, especially in children [4, 5]. In 2016, the new WHO classification has classified *t*(6; 11) renal cell carcinoma and Xp11.2 translocation/TFE3 gene fusion-related renal cell carcinoma into MIT family translocation renal cell carcinoma, referred to as Xp11.2 translocation renal cell carcinoma. Comparing to other subtypes of RCC, this neoplasm has more aggressive clinicopathologic features at diagnosis and worse prognosis [3, 5, 6]. To better predict the risk of disease reoccurrence and death, it is important to conduct prognostic studies to identify potential preoperative risk factors for disease progression and death which might help to guide interventions in the future. Moreover, prognostic research on adult patients should be especially encouraged due to at least three reasons: first, as a rare disease which mainly affects children, data for adult patients is scarce right now [4]; second, this disease manifests with a more aggressive behavior in adults than in children, suggesting possibly different prognostic features in adults [3]; third, prior prognostic studies, which revealed several possible risk factors, such as neutrophil-to-lymphocyte ratio (NLR), C-reactive protein/albumin ratio (CRP/Alb ratio), platelet-to-lymphocyte ratio (PLR), tumor stage, and inferior vena cava tumor thrombosis, included both pediatric and adult patients for analysis which might mask the factors specific for adults [6, 7]. Therefore, it would be of importance to identify novel prognostic factors in adult XP11.2 translocation RCC patients.

The article "Xp11.2 Translocation Renal Cell Carcinoma: Clinical Characteristics and Potential Prognostic Predictors" was published in 2021. Journal: Dis Markers.

Herein, we embarked on a study to explore the clinical characteristics and potential prognostic predictors for adult patients with newly diagnosed XP11.2 translocation RCC.

## 2. Patients and Methods

### 2.1. Patients

Between April 2010 and March 2020, 24 patients diagnosed with XP11.2 translocation RCC after percutaneous renal mass biopsy or nephrectomy (radical or partial) at Peking Union Medical College Hospital (PUMCH) were recruited. Clinical information was retrieved from medical records from the department of urology. Pathological reports were carefully reviewed, and TFE3 immunohistochemistry staining results were reconfirmed. The inclusion criteria were (1) typical morphological pattern plus moderate-to-strong nuclear positivity with TFE3 immunohistochemistry staining results; (2) complete blood laboratory tests including blood routine test, blood biochemistry tests, and coagulation test within one week before biopsy or nephrectomy; and (3) adult patients defined as 16 years or older. The exclusion criteria were (1) pregnant women, (2) <16 years old, and (3) with other inflammatory disease or a second tumor. This study was performed in accordance with relevant guidelines and regulations and was approved by the PUMCH Ethics Committee. Informed consent was achieved from all patients for the utilization of their medical records.

Demographic, clinical, laboratory, and treatment-related data, including age at the time of diagnosis, gender, symptoms at presentation, serological results, radiological findings, and treatment strategies, were documented. Preoperative neutrophil count, lymphocyte count, platelet count, hemoglobin level, C-reactive protein (CRP) level, albumin level, lactic dehydrogenase (LDH) level, and fibrinogen (Fbg) level were collected. Possible prognostic factors such as NLR (neutrophil-to-lymphocyte ratio), PLR (platelet-to-lymphocyte ratio), and CRP/Alb (CRP/albumin ratio) were calculated [6]. Presence of tumor thrombus of inferior vena cava (IVC), lymph node metastasis, and distant metastasis were confirmed from radiological examinations.

### 2.2. Follow-Up

Patient follow-up was conducted via interviews at an outpatient clinic, telephone contacts, letters, and analyses of information documented in the hospital database. Patients were followed until March 2020, and follow-up results were analyzed by two independent urologists to determine progression. Progression was defined as tumor relapse, enlargement of tumor mass, or presence of new metastatic lesions. Progression-free survival (PFS) was defined as the time from diagnosis to disease progression or death from any cause. Overall survival (OS) was defined as the time from diagnosis to death from any cause.

### 2.3. Statistical Analysis

Statistical analysis was performed using SPSS 13.0 (SPSS Inc., Chicago, IL). Possible risk factors for progression-free survival and overall survival were firstly scanned with chi-square tests (for categorical covariates) and *t*-tests (for continuous covariates) to compare patients who suffered from progression (or death) and who did not. NLR, PLR, and CRP/Alb were transcoded into categorical variables with cutoff values set at 2.45, 140, and 0.083, respectively, according to a prior study [6]. Variables with *p* < 0.10 revealed by univariate comparison were further analyzed with multivariate Cox regression. A stepwise regression strategy with a backward method (criteria for entry and removal of variables were *p* < 0.05 and *p* > 0.10) was utilized with 1 variable eliminated at a time. Parameters with *p* < 0.05 were considered to represent independent predictors of PFS or OS. Dichotomous variables which showed to be independent risk factors were further analyzed by the Kaplan-Meier method for depicting survival curves using log-rank tests for comparison. For the convenience of survival curve depicting, continuous variables revealed as independent risk factors via multivariate Cox regression were transcoded into dichotomous variables with cutoff values set according to ROC curve analysis.

The article "Xp11.2 Translocation Renal Cell Carcinoma: Clinical Characteristics and Potential Prognostic Predictors" was published in 2021. Journal: Dis Markers.

## 3. Results

### 3.1. Patient Characteristics

A total of 4958 cases of adult RCC were diagnosed in the past ten years at our center. Among them, 24 patients were diagnosed with XP 11.2 translocation RCC (overall proportion 0.48%).  Table 1 outlines clinical characteristics of these 24 patients, including 12 (50.0%) males and 12 (50.0%) females. The median age at diagnosis of XP 11.2 translocation RCC was 32 years (range, 16-73 years). At the time of diagnosis, eleven patients (45.8%) were symptomatic while 13 patients (54.2%) were asymptomatic. Tumors were found on 15 right kidneys (62.5%) and 9 left kidneys (37.5%) with a mean tumor size (maximum diameter) of 8.05 ± 5.13 cm. A large proportion of patients showed evidence of advanced stage at the time point of diagnosis: 45.8% patients with lymph node metastasis, 25% patients with distant metastasis, and 20.8% patients with tumor thrombus of IVC. Two patients did not receive further surgery after percutaneous renal mass biopsy-proven diagnosis. Twenty-two patients underwent nephrectomy (radical 16/22 or partial 6/22). After obtaining pathology, patients with tumors of advanced stage received additional treatment. One patient with IVC tumor thrombus received interleukin-1 therapy and died 56 months after operation. The other patients received targeted drug therapy (sunitinib or sorafenib). After a mean follow-up of 35.7 months, a total of nine patients had a progression of disease, and seven patients died. The estimated 3-year progression-free survival was 66% and 3-year OS was 88.1%.

### 3.2. Risk Factors Associated with Progression

With univariate analysis (Table 2), higher C-reactive protein-to-albumin ratio (CRP/Alb) (*p* = 0.028), higher baseline fibrinogen (*p* = 0.006), and presence of distant metastasis (*p* = 0.007) were associated with progression of the disease. All of them, with a *p* value less than 0.10, entered the multivariate Cox regression with a backward stepwise method. At the last step (Table 2), the baseline fibrinogen level (HR 5.761; 95% confidence interval (CI) 1.958-16.949; *p* = 0.001) was identified as the only independent risk factor for PFS.

### 3.3. Risk Factors Associated with Overall Survival

Univariate analysis revealed four candidates (*p* < 0.10) for further multivariate regression: CRP/Alb (*p* = 0.053), preoperative fibrinogen (*p* = 0.014), tumor thrombus of IVC (*p* = 0.088), and distant metastasis (*p* = 0.020). Among them, fibrinogen level and presence of distant metastasis were considered statistically significant risk factors (*p* < 0.05) for death using univariate scanning. After multivariate analysis, fibrinogen level (HR 2.954; 95% CI 1.011-8.629; *p* = 0.048) and distant metastasis (HR 12.287; 95% CI 1.083-139.409; *p* = 0.043) were identified as independent risk factors for survival.

The article "Xp11.2 Translocation Renal Cell Carcinoma: Clinical Characteristics and Potential Prognostic Predictors" was published in 2021. Journal: Dis Markers.

### 3.4. Survival Curves

According to ROC curve analysis, the area under the curve (AUC) value of preoperative fibrinogen of overall survival was 0.861 (*p* = 0.006). The optimal cutoff value for fibrinogen was 3.84 g/L. Fibrinogen (Fbg), a continuous variable, was then transcoded into a dichotomous variable (Fbg ≥ 3.84 g/L versus Fbg < 3.84 g/L) for survival curve depicting.  Figure 1(a) shows a significant difference of PFS (*p* < 0.001) between patients with and without elevated (≥3.84 g/L) fibrinogen: patients with baseline Fbg < 3.84 g/L did not reach the median PFS of patients with elevated fibrinogen (34 months).  Figure 1(b) reveals a significant difference of OS (*p* = 0.0417) between these two groups: median survival 56 months for patients with Fbg < 3.84 g/L versus 48 months for patients with Fbg ≥ 3.84 g/L.

Presence of distant metastasis, a dichotomous variable which was shown to be a risk factor for progression with univariate analysis and an independent risk factor for overall survival with multivariate analysis, was further used to delineate survival curves (Figure 2). Significant difference was noted for PFS (*p* = 0.0082): median survival for patients without distant metastasis was 46 months comparing to 22 months in patients with distant metastasis (Figure 2(a)).  Figure 2(b) shows a significant difference of OS for patients with and without distant metastasis (median survival 48 months versus 56 months, *p* = 0.025).

## 4. Discussion

XP11.2 translocation RCC accounts for 20-40% of pediatric RCC and only 0.72-1.6% of adult RCC [5, 8–10]. This subtype of RCC in adults requires special attention and more intensive studies for its rarity, aggressiveness in nature, and possible different treatment options (e.g., mTOR inhibitors or VEGF-targeted agents) [3, 8, 11, 12]. This single-center, retrospective study identified an overall incidence of 0.48% for XP11.2 translocation RCC out of all adult RCCs based on a ten-year data. This result was consistent with another Asian cohort (0.72% in Korea) which further demonstrated the rarity of this disease in adults [5]. Although a prior meta-analysis suggested a female gender predominance in adult XP11.2 translocation RCC, possibly due to its X chromosome-related nature, our study found an equal gender distribution as observed in children which might be explained by the absence of translocation on the Barr body (inactive X chromosome) or by the relatively small number of patients enrolled [8]. Moreover, consistent with previous reports and for unknown reasons, higher prevalence on the right side was observed in our cohort [7, 13].

The article "Xp11.2 Translocation Renal Cell Carcinoma: Clinical Characteristics and Potential Prognostic Predictors" was published in 2021. Journal: Dis Markers.

Several attempts have been made to investigate the possible risk factors for survival which suggested several possible risk factors as NLR, CRP/Alb, PLR, and tumor thrombosis of IVC and tumor stage [6, 7]. However, disparities are noticed in different studies, and these factors have never been externally validated. Moreover, these studies enrolled both children and adult patients which might hinder the accuracy of the prediction models as children present relatively indolent disease course [3]. This study, according to our limited knowledge, is one of the first endeavors to validate those previously reported prognostic factors and to explore novel potential risk factors in adult patients with XP11.2 translocation RCC. In this study, previously reported risk factors such as CRP/Alb and tumor thrombosis of IVC showed statistical significance or borderline significance (Tables 2 and 3) with univariate analysis [6, 7]; and distant metastasis, a parameter reflecting tumor stage, showed to be an independent risk factor for OS with multivariate analysis. Moreover, preoperative plasma fibrinogen, a parameter routinely examined preoperatively but never tested for risk stratification in XP11.2 translocation RCC, was reported to be an independent risk factor for both PFS and OS.

Elevated fibrinogen levels have been linked to poor outcomes in many types of cancer, including kidney malignancies [14–18]. However, its role in predicting survival in XP11.2 translocation RCC has not been well illuminated. In this retrospective study, we not only demonstrated its independent nature to predict progression but also suggested a crucial role to predict overall survival. There have been several theories to explain the association between fibrinogen and outcomes of malignancies: first, a high fibrinogen level might be a reflection of tumor induced systemic inflammatory response [19]; second, fibrinogen can be endogenously synthesized by tumor cells and in return facilitates tumor growth and metastasis [17, 20]; third, fibrinogen could activate tumor cell adhesion with platelets to form a dense fibrin “protective” layer around tumor cells from natural killer cells [21]. Aside from these common pathways, there might be two other distinct mechanisms to clarify the association between fibrinogen and outcomes of XP11.2 translocation RCC, a tumor which has been demonstrated to involve VEGF and mTOR pathways [11, 12]: as an extracellular matrix element, fibrinogen could regulate growth of cancer cells by binding to VEGF [22]; alternatively, fibrinogen may promote cell motility by inducing epithelial-mesenchymal transition via the p-AKT/p-mTOR pathway [23]. These mechanisms may underline the link between fibrinogen and this unique subtype of RCC and explain the strong association found in this study.

The article "Xp11.2 Translocation Renal Cell Carcinoma: Clinical Characteristics and Potential Prognostic Predictors" was published in 2021. Journal: Dis Markers.

Our study has limitations: first of all, due to the scarcity of cases, the sample size in this paper is limited. This may affect the strength of the conclusion to a certain extent, which needs to be verified in future research; second, the TFE3 break-apart FISH analysis was not done for this cohort of patients. Although TFE3 immunohistochemistry was also an accurate tool for diagnosis which had been accepted by prior studies, we still utilized TFE3 immunohistochemistry stain as our inclusion criteria [3, 6]. Third, the results of this study were not externally validated, and future work focusing on the role of fibrinogen in XP11.2 translocation RCC might be helpful.

In conclusion, relatively high CRP/Alb ratios, fibrinogen, and distant metastasis are associated with a poor prognosis of Xp11.2 tRCC patients; among them, preoperative plasma fibrinogen, a routinely tested parameter before surgery, independently predicts the progression of Xp11.2 tRCC and may help identify patients with worse progression or death risk.

## Figures and Tables

**Figure 1:** Survival curves of PFS (Figure 1(a)) and OS (Figure 1(b)) with a cutoff point of fibrinogen at 3.84 g/L.

**Figure 2:** Survival curves of PFS (Figure 2(a)) and OS (Figure 2(b)) for patients with and without distant metastasis.

**Table 1:** Clinical characteristics of patients with Xp11.2 translocation RCC.

	Value	%
Gender		
Male	12	50%
Female	12	50%
Age (year)	42.7 ± 14.9	
Symptoms at onset		
Symptomatic	11	45.80%
Asymptomatic	13	54.20%
Location		
Right	15	62.50%
Left	9	37.50%
Tumor size (cm)	8.05 ± 5.13	
Lymph node metastasis		
Positive	11	45.80%
Negative	13	54.20%
Distant metastasis		
Positive	6	25.00%
Negative	18	75.00%
Tumor thrombus of IVC		
Positive	5	20.80%
Negative	19	79.20%
Surgical treatment		
No surgery	2	8.30%
Partial	6	25.00%
Radical	16	66.70%
Additional treatment		
Interleukin-1	6	25.00%
Targeted drug	10	41.67%

RCC: renal cell carcinoma; IVC: inferior vena cava.

**Table 2:** Risk factors for disease progression in patients with Xp11.2 translocation RCC.

	Univariate analysis			Multivariate Cox regression (last step)	
	Progression	No progression	*p*	HR (95% CI)	*p*
Gender, male (*n*)	4/9	8/15	0.673		
Age (year)	46.6 ± 17.7	40.4 ± 13.2	0.340		
Symptomatic patient (*n*)	6/9	5/15	0.113		
Right side (*n*)	5/9	4/15	0.157		
Tumor size (cm)	9.13 ± 5.82	7.40 ± 4.76	0.435		
NLR > 2.45	7/9	8/15	0.231		
PLR > 140	4/9	9/15	0.459		
CRP/Alb > 0.083	5/9	2/15	0.028		
LDH (U/L)	255.3 ± 101.8	201.0 ± 104.8	0.227		
Hemoglobin (g/L)	123.2 ± 23.3	132.8 ± 20.7	0.306		
Fbg (g/L)	3.95 ± 1.04	2.69 ± 0.47	0.006	5.761 (1.958-16.949)	0.001
Tumor thrombus of IVC	3/9	2/15	0.243		
Lymph node metastasis	6/9	5/15	0.113		
Distant metastasis	5/9	1/15	0.007		
Radical surgery^∗^	5/7	11/15	0.926		
Additional treatment					
Targeted drug only	2/9	0/15			
Surgery only	1/9	7/15			
Surgery+interleukin-1	3/9	3/15			
Surgery+targeted drug	3/9	5/15			

NLR: neutrophil-to-lymphocyte ratio; PLR: platelet-to-lymphocyte ratio; CRP/Alb: C-reactive protein/albumin ratio; LDH: lactic dehydrogenase; Fbg: fibrinogen; IVC: inferior vena cava. ^∗^For patients who had surgical treatment, *n* = 22.

The article "Xp11.2 Translocation Renal Cell Carcinoma: Clinical Characteristics and Potential Prognostic Predictors" was published in 2021. Journal: Dis Markers.

**Table 3:** Risk factors for death in patients with Xp11.2 translocation RCC.

	Univariate analysis			Multivariate Cox regression (last step)	
	Death	No death	*p*	HR (95% CI)	*p*
Gender, male (*n*)	4/7	8/17	0.653		
Age (year)	46.4 ± 19.7	41.2 ± 12.9	0.446		
Symptomatic patient (*n*)	4/7	7/17	0.476		
Right side (*n*)	4/7	5/17	0.202		
Tumor size (cm)	8.87 ± 6.47	7.71 ± 4.66	0.626		
NLR > 2.45	5/7	10/17	0.562		
PLR > 140	2/7	11/17	0.106		
CRP/Alb > 0.083	4/7	3/17	0.053		
LDH (U/L)	239.9 ± 107.8	213.8 ± 106.1	0.591		
Hemoglobin (g/L)	122.1 ± 23.2	132.1 ± 21.1	0.317		
Fbg (g/L)	4.16 ± 1.10	2.76 ± 0.47	0.014	2.954 (1.011-8.629)	0.048
Tumor thrombus of IVC	3/7	2/17	0.088		
Lymph node metastasis	5/7	6/17	0.106		
Distant metastasis	4/7	2/17	0.020	12.287 (1.083-139.409)	0.043
Radical surgery^∗^	4/6	12/16	0.696		
Additional treatment					
Targeted drug only	1/7	1/17			
Surgery only	1/7	7/17			
Surgery+interleukin-1	2/7	4/17			
Surgery+targeted drug	3/7	5/17			

NLR: neutrophil-to-lymphocyte ratio; PLR: platelet-to-lymphocyte ratio; CRP/Alb: C-reactive protein/albumin ratio; Fbg: fibrinogen; LDH: lactic dehydrogenase. ^∗^For patients who had surgical treatment, *n* = 22.

## Data Availability

The data used to support the findings of this study are included within the article.

## References

[1] Argani P., Ladanyi M. (2005). Translocation carcinomas of the kidney. *Clinics in Laboratory Medicine*.

[2] Ellis C. L., Eble J. N., Subhawong A. P. (2014). Clinical heterogeneity of Xp11 translocation renal cell carcinoma: impact of fusion subtype, age, and stage. *Modern Pathology*.

The article "Xp11.2 Translocation Renal Cell Carcinoma: Clinical Characteristics and Potential Prognostic Predictors" was published in 2021. Journal: Dis Markers.

[3] Kuthi L., Somorácz Á., Micsik T. (2020). Clinicopathological findings on 28 cases with XP11.2 renal cell carcinoma. *Pathology Oncology Research*.

[4] Argani P., Lal P., Hutchinson B., Lui M. Y., Reuter V. E., Ladanyi M. (2003). Aberrant nuclear immunoreactivity for TFE3 in neoplasms with TFE3 gene fusions: a sensitive and specific immunohistochemical assay. *The American Journal of Surgical Pathology*.

[5] Choo M. S., Jeong C. W., Song C. (2017). Clinicopathologic characteristics and prognosis of Xp11.2 translocation renal cell carcinoma: multicenter, propensity score matching analysis. *Clinical Genitourinary Cancer*.

[6] Agizamhan S., Qu F., Liu N. (2018). Preoperative neutrophil-to-lymphocyte ratio predicts the surgical outcome of Xp11.2 translocation/TFE3 renal cell carcinoma patients. *BMC Urology*.

[7] Liu N., Wang Z., Gan W. (2016). Renal cell carcinoma associated with Xp11.2 translocation/TFE3 gene fusions: clinical features, treatments and prognosis. *PLoS One*.

[8] Cheng X., Gan W., Zhang G., Li X., Guo H. (2016). Clinical characteristics of XP11.2 translocation/TFE3 gene fusion renal cell carcinoma: a systematic review and meta-analysis of observational studies. *BMC Urology*.

[9] Komai Y., Fujiwara M., Fujii Y. (2009). Adult Xp11 translocation renal cell carcinoma diagnosed by cytogenetics and immunohistochemistry. *Clinical Cancer Research*.

[10] Qu Y., Gu C., Wang H. (2016). Diagnosis of adults Xp11.2 translocation renal cell carcinoma by immunohistochemistry and FISH assays: clinicopathological data from ethnic Chinese population. *Scientific Reports*.

[11] Malouf G. G., Camparo P., Oudard S. (2010). Targeted agents in metastatic Xp11 translocation/ TFE3 gene fusion renal cell carcinoma (RCC): a report from the Juvenile RCC Network. *Annals of Oncology*.

[12] Choueiri T. K., Lim Z. D., Hirsch M. S. (2010). Vascular endothelial growth factor-targeted therapy for the treatment of adult metastatic Xp11.2 translocation renal cell carcinoma. *Cancer*.

[13] Hirobe M., Masumori N., Tanaka T. (2016). Clinicopathological characteristics of Xp11.2 translocation renal cell carcinoma in adolescents and adults: Diagnosis using immunostaining of transcription factor E3 and fluorescence in situ hybridization analysis. *International Journal of Urology*.

[14] Takeuchi H., Ikeuchi S., Kitagawa Y. (2007). Pretreatment plasma fibrinogen level correlates with tumor progression and metastasis in patients with squamous cell carcinoma of the esophagus. *Journal of Gastroenterology and Hepatology*.

[15] Palumbo J. S., Kombrinck K. W., Drew A. F. (2000). Fibrinogen is an important determinant of the metastatic potential of circulating tumor cells. *Blood*.

The article "Xp11.2 Translocation Renal Cell Carcinoma: Clinical Characteristics and Potential Prognostic Predictors" was published in 2021. Journal: Dis Markers.

[16] Fan S., Guan Y., Zhao G., An G. (2018). Association between plasma fibrinogen and survival in patients with small-cell lung carcinoma. *Thorac Cancer*.

[17] Tian Y., Hong M., Jing S. (2017). Clinical and prognostic effect of plasma fibrinogen in renal cell carcinoma: a meta-analysis. *BioMed Research International*.

[18] He X., Huang T., Xue Y. (2019). Association of preoperative plasma D-dimmer and fibrinogen and renal cell carcinoma outcome. *Journal of Cancer*.

[19] Lip G. Y., Chin B. S., Blann A. D. (2002). Cancer and the prothrombotic state. *The Lancet Oncology*.

[20] Simpson-Haidaris P. J., Rybarczyk B. (2001). Tumors and fibrinogen. The role of fibrinogen as an extracellular matrix protein. *Annals of the New York Academy of Sciences*.

[21] Zheng S., Shen J., Jiao Y. (2009). Platelets and fibrinogen facilitate each other in protecting tumor cells from natural killer cytotoxicity. *Cancer Science*.

[22] Sahni A., Francis C. W. (2000). Vascular endothelial growth factor binds to fibrinogen and fibrin and stimulates endothelial cell proliferation. *Blood*.

[23] Zhang F., Wang Y., Sun P. (2017). Fibrinogen promotes malignant biological tumor behavior involving epithelial-mesenchymal transition via the p-AKT/p-mTOR pathway in esophageal squamous cell carcinoma. *Journal of Cancer Research and Clinical Oncology*.

